The article "Application of Touching Combined with Intelligent Interaction of Voice and Rhythm in Nursing Care of Newborns with Feeding Intolerance and Its Influence on Quality of Life" was retracted in 2023. Reasons: unreliable results or conclusions; concerns about the data; concerns about the peer review; concerns about the citations.

# Application of Touching Combined with Intelligent Interaction of Voice and Rhythm in Nursing Care of Newborns with Feeding Intolerance and Its Influence on Quality of Life

**DOI:** 10.1155/2022/4747337

**Published:** 2022-04-01

**Authors:** Liang Shan, Juan Li, Ping Rong Yang, Hua De Jin, Jiang Guo, Hong Xiao

**Affiliations:** Panzhihua Central Hospital Paediatrics, 617000, China

## Abstract

**Objective:**

To explore the application of touching combined with intelligent interaction of voice and rhythm in the nursing of neonatal feeding intolerance and its effect on the quality of life.

**Methods:**

A total of 140 newborns with feeding intolerance treated in our hospital from April 2019 to April 2021 were selected. The patients were randomly divided into two groups: the control group and the study group. The control group received touch nursing and the study group received touch combined with intelligent interactive nursing mode of voice, music, and rhythm. The general data, feeding performance, feeding process, growth and development, feeding intolerance, total intestinal feeding, jaundice duration, hospital stay, and quality of life scores were compared between the two groups.

**Results:**

First of all, we compared the general data of the two groups. There was no significant difference in gestational age, sex, mode of delivery, birth weight, head circumference, body length, Apgar score, and other general data between the two groups. Second, we compared the feeding performance of the two groups. Before nursing, there was no significant difference between the two groups (*P* > 0.05). After nursing, the feeding rate, milk intake ratio, and proficiency of the two groups increased, and the comparison between the two groups. The feeding rate, milk intake ratio, and proficiency of the study group were better than those of the control group. In terms of the feeding process of the two groups, the days of oral feeding, complete import feeding, feeding conversion, and indwelling gastric tube in the study group were lower than those in the control group (*P* < 0.05). In terms of the growth and development of the two groups, the recovery time of birth weight in the study group was lower than that in the control group, and the growth of body weight, length, and head circumference at 14 days in the study group was higher than those in the control group. The feeding intolerance, the duration of jaundice, and the days of hospitalization in the study group were lower than those in the control group (*P* < 0.05). Moreover, the feeding intolerance, the duration of jaundice, and the days of hospitalization in the study group were lower than those in the control group (*P* < 0.05). Finally, we compared the scores of qualities of life between the two groups. The physiological function, psychological function, and social function of the study group were lower than those of the control group (*P* < 0.05). The physiological function, psychological function, and social function of the study group were lower than those of the control group (*P* < 0.05).

The article "Application of Touching Combined with Intelligent Interaction of Voice and Rhythm in Nursing Care of Newborns with Feeding Intolerance and Its Influence on Quality of Life" was retracted in 2023. Reasons: unreliable results or conclusions; concerns about the data; concerns about the peer review; concerns about the citations.

**Conclusion:**

The application of touching combined with phonetic rhythm intelligent interaction technology in the nursing of neonatal feeding intolerance can promote the faster development and maturity of neonatal gastrointestinal function, improve gastrointestinal motility, shorten the time of parenteral nutrition in newborns, achieve total enteral feeding faster, and promote neonatal growth and development, so as to shorten the duration of hospitalization, improve the tolerance of neonatal gastrointestinal feeding, and improve the quality of life.

## 1. Introduction

Neonatal feeding difficulty, that is, neonatal feeding intolerance, is a group of symptoms caused by gastrointestinal dysfunction induced by a variety of disease factors, such as vomiting, gastric retention, and abdominal distension [1]. Once neonatal feeding difficulties occur, it will lead to gastrointestinal nutrition supply disorders and delay the rehabilitation of basic diseases, eventually prolong the length of stay and reduce the chances of neonatal survival and increase the psychological and economic burden of society and families [1]. Premature infants, intrauterine distress, ventricular rest, severe infection, and other disease factors are prone to lead to neonatal feeding intolerance. The physiological characteristics of insufficient gastric volume, weak gastrointestinal peristalsis, poor sucking ability, relaxation of cardiac sphincter, and insufficient gastric motility can easily lead to feeding intolerance symptoms such as frequent vomiting, gastric retention, abdominal distension, and lack of milk [2]. The improvement of gastrointestinal motility is the key factor to improve neonatal feeding tolerance. Promoting neonatal gastrointestinal motility can improve the success rate of neonatal enteral feeding. Modern medicine is often treated with western medicine, such as injection of erythromycin oral bifidobacterium, domperidone, and other gastrointestinal motility drugs as well as nondrug therapy, such as nonnutritional sucking and neonatal massage [1]. Touching refers to the orderly and skillful massage of newborns under the guidance of science, so that a large number of mild and good stimuli are transmitted to the central nervous system through skin receptors, thus producing positive physiological effects [2]. Touching originated in 1881, was introduced into China in 1995, and was recognized and recommended by Pediatrics Branch of Chinese Medical Association, Perinatal Medical Association, and Chinese Nursing Association in 2001 [3]. Touching can be transmitted to the brain along the medulla oblongata through the tactile receptors on the body surface, and messages are sent from the brain to excite the vagus nerve, thus increasing gastrointestinal peristalsis and gastrointestinal endocrine hormone activities, promoting the digestion and absorption of nutrients in infants [4]. However, neonatal gastric volume is insufficient, gastrointestinal emptying capacity is weak, emptying time is long, drug injection and oral drug feeding are inconvenient, touching is not systematic, and treatment often cannot achieve the expected effect.

The article "Application of Touching Combined with Intelligent Interaction of Voice and Rhythm in Nursing Care of Newborns with Feeding Intolerance and Its Influence on Quality of Life" was retracted in 2023. Reasons: unreliable results or conclusions; concerns about the data; concerns about the peer review; concerns about the citations.

In recent years, the field of research and development of artificial intelligence (AI) chips is becoming more and more perfect. Since 2015, the State Council of China put forward the guidance for upgrading the horizontal connection of the industry with “Internet +” as the core, and since the Robot Industry Development Plan was released in 2016, great progress has been made in artificial intelligence (AI) technology in China, and intelligent products based on AI have come out one after another. The main areas involved are the household, retail, transportation, medical care, education, and so on [4]. With the development of society, intelligent automation system is gradually applied to the service industry. At present, voice interaction equipment is one of the products of the intelligent era, and academia and industry continue to invest in the field of voice interaction, fighting for a leading position [5]. The essence of AI of speech music and rhythm is natural language processing. It is not difficult to imagine that in the future life; intelligent robots will become an indispensable member of human life [6]. Even medical staff who have not been trained can use this technology to carry out nursing operation on their own. Through this technology, we can intelligently adjust the rhythm of speech and stimulate the sensory system of newborns, so as to promote growth [7]. In the past, there were many clinical reports on the application of touch nursing in neonatal feeding intolerance [8], but the combined report was few. This study focuses on the application of touching combined with phonetic rhythm intelligent interaction in neonatal feeding intolerance nursing and its impact on the quality of life.

## 2. Patients and Methods

### 2.1. Patient Information

A total of 140 newborns with feeding intolerance treated in our hospital from April 2019 to April 2021 were selected. The patients were randomly divided into two groups: the control group and the study group. The control group received touch nursing and the study group received touch combined with intelligent interactive nursing mode of voice, music, and rhythm. In the control group, the gestational age was 26-42 weeks, and in the study group, the gestational age was 26-41 weeks. There was no statistical significance in the general data of the two groups (see Table 1). This study was approved by the Medical Ethics Association of our hospital, and all patients signed informed consent.

The article "Application of Touching Combined with Intelligent Interaction of Voice and Rhythm in Nursing Care of Newborns with Feeding Intolerance and Its Influence on Quality of Life" was retracted in 2023. Reasons: unreliable results or conclusions; concerns about the data; concerns about the peer review; concerns about the citations.

Diagnostic criteria: according to the diagnostic criteria of neonatal feeding intolerance put forward by Huang Ying in 2000, the diagnostic criteria of neonatal feeding difficulties were as follows: (1) frequent vomiting (2-3 times per day), (2) no increase or decrease in milk volume (>3 days), and (3) gastric retention (retention > 1 stroke 3 of the previous feeding volume).

The inclusion criteria were as follows: (1) newborns with gestational age of 26-42 weeks; (2) accorded with the diagnosis of feeding intolerance.

Exclusion criteria: (1) complicated with congenital malformation; (2) neonatal necrotizing enterocolitis, respiratory and circulatory failure, and genetic metabolic diseases; (3) complicated with severe intrauterine distress and ventricular dyspnea; (4) severe skin damage and infection.

Withdrawal criteria: (1) complicated with serious complications (such as intracranial hemorrhage, pulmonary hemorrhage, gastrointestinal hemorrhage, and NEC); (2) drug intolerance or serious adverse events related to treatment regimen; (3) researchers believe that continuing the trial may cause damage to the subjects; (4) family members of children do not cooperate with treatment; (5) patients discharged from hospital midway to finish treatment due to economic and other reasons.

### 2.2. Nursing Method

Both groups received routine treatment, diagnosed and treated according to the guidelines of neonatal management. During the treatment of feeding intolerance, nonnutritive sucking of nonperforated rubber nipples was given for 10 minutes, plus low-dose erythromycin (5 mg/kg/, qd, intravenous infusion with infusion pump within 1 hour for 3-5 days).

The control group received touch nursing intervention, the newborn was placed on the radiation table, and the radiation station was preheated in advance. The temperature was set at 34-36°C and connected with ECG monitoring. Using the formal international standard method [31], newborns exposed the whole body and massaged sequentially from head, face, chest, abdomen, upper limbs, palms, fingers, lower limbs, soles, toes, and back. Under the condition that the newborn was quiet, awake, and without hunger or fatigue, the touch was given after bathing, and the first touch was from 5 min. If the newborn showed no symptoms of discomfort, it would prolong to 10 min. The operators are senior NICU nurses who were trained and qualified by the baby touch system. Cutting the nails before touching to avoid scratching. Wash the hands in seven steps and warm the hands and apply emollient oil to lubricate your hands. During the operation, the operator made gentle eye contact and cordial verbal communication with the newborn and closely observed the vital signs and reactions of the newborn. If the blood oxygen saturation dropped below 90%, lips cyanosis, shortness of breath, etc., should immediately stop touching and give oxygen inhalation. When the newborn cried, did not cooperate, muscle tension, vomiting should stop touching. Try to keep the surrounding environment quiet during touching to avoid intrusive operation.

The article "Application of Touching Combined with Intelligent Interaction of Voice and Rhythm in Nursing Care of Newborns with Feeding Intolerance and Its Influence on Quality of Life" was retracted in 2023. Reasons: unreliable results or conclusions; concerns about the data; concerns about the peer review; concerns about the citations.

On the basis of the control group, combined with the intelligent interaction technology of voice rhythm, the specific measures of the study group were as follows: the researcher entered the maternal ward to collect voice rhythm. Researchers needed to communicate and explain to pregnant women and other family members and obtain their cooperation. The content of phonetic rhythm was the children's songs, short stories, or gentle words that parturient often play or hum for the fetus during pregnancy. Before recording, edit the speaking or singing content into a paper version, let the pregnant woman practice the humming or saying content several times according to the paper content, and guide its tone, intonation, or rhythm, and then record it with a recorder. After recording, the audio editing software was used to reduce noise, no vibrato, and other processing. 5 min began to play MSS before the newborn was breast-fed, and the playback time was 15 min each time. The specific method was as follows: put the recorder into the warm box, the distance from the infant's ears was about 20 cm, to start 5 min before breast-feeding, the sound intensity is 50-55 dB, and play it once at 09 : 00, 12 : 00, 15 : 00, and 18 : 00 every day, each time 15 min. When playing the recording, it was necessary to control the sound intensity of the external environment not to exceed the 65 dB. Avoid invasive operations such as venipuncture and blood sampling. In the course of intervention, if the blood oxygen saturation decreased, heart rate reduced, apnea, vomiting, and other conditions immediately stopped the intervention.

### 2.3. Observation Indicators

#### 2.3.1. General Information

Access to neonatal-related case data, record all selected people's gestational age, sex, mode of delivery, birth weight, head circumference, body length, Apgar score, and other general data.

The article "Application of Touching Combined with Intelligent Interaction of Voice and Rhythm in Nursing Care of Newborns with Feeding Intolerance and Its Influence on Quality of Life" was retracted in 2023. Reasons: unreliable results or conclusions; concerns about the data; concerns about the peer review; concerns about the citations.

#### 2.3.2. Feeding Performance

The feeding rate, milk intake ratio, and proficiency of the two groups before and after nursing were calculated. The feeding activities of newborns at 09 : 00, 12 : 00, 15 : 00, and 18 : 00 were observed, and the feeding performance in the four feeding activities was recorded and averaged.

#### 2.3.3. Feeding Process

Feeding process: the beginning of oral feeding, the corresponding gestational age at complete oral feeding, the conversion time from oral feeding to complete oral feeding (days), and the time of indwelling gastric tube (days). The beginning of oral feeding refers to the first oral milk intake ≥5 ml/times, and complete oral feeding refers to oral milk intake reaching 120 ml/kg. d-1 and gastric tube removal time ≥48 hours.

#### 2.3.4. Growth and Development

Growth and development index: the time of recovery to birth weight (days) and the increase of body mass (g), body length (cm), and head circumference (cm) on the 14th day in hospital were observed and recorded.

#### 2.3.5. Feeding Intolerance, Reaching Whole Intestinal Feeding, Duration of Jaundice, and Length of Stay

The feeding intolerance, the total enteral feeding, the duration of jaundice, and the days of hospitalization were calculated between the two groups. Feeding intolerance: any of the following conditions is diagnosed as feeding intolerance: vomiting: ≥3 times/day, abdominal distension: increased abdominal circumference > 1.5 cm/day with intestinal type, gastric retention: retention volume > 1 × 3 of the last feeding volume, occurrence ≥ 3 times/day, brown gastric contents, positive fecal occult blood, apnea, and bradycardia increased by more than 50% compared with the previous day.

#### 2.3.6. Quality of Life Scale

The quality of life scale [9] consists of three subscales, including physiological, psychological, and social functions, with a total of 29 items. The Cronbach's *α* coefficient of the scale is 0.79-0.91. The scale was scored by 1-5 grades. The lower the score, the higher the satisfaction.

### 2.4. Statistical Analysis

Mean ± standard deviation was used for statistical description, *t*-test was used for counting data, *χ*^2^ test was used for counting data, rank sum test was used for grade data, and percentage was used to describe and analyze the data. Statistical software SPSS21.0, *P* < 0.05 indicates that the difference is statistically significant and *P* less than 0.01 means that the higher difference is statistically significant.

The article "Application of Touching Combined with Intelligent Interaction of Voice and Rhythm in Nursing Care of Newborns with Feeding Intolerance and Its Influence on Quality of Life" was retracted in 2023. Reasons: unreliable results or conclusions; concerns about the data; concerns about the peer review; concerns about the citations.

## 3. Results

### 3.1. Comparison of General Data of Two Groups of Patients

First of all, we compared the general data of the two groups. There was no significant difference in gestational age, sex, mode of delivery, birth weight, head circumference, body length, Apgar score, and other general data between the two groups (*P* > 0.05). All the data are presented in Table 1.

### 3.2. Comparison of Feeding Performance

Second, we compared the feeding performance of the two groups; before nursing, there was no significant difference between the two groups (*P* > 0.05). After nursing, the feeding rate, milk intake ratio, and proficiency of the two groups increased; the feeding rate, milk intake ratio, and proficiency of the study group were better than those of the control group; and the difference was statistically significant (*P* < 0.05). All the data results are shown in Figures 1(a) and 1(b).

### 3.3. Comparison of Feeding Process

Next, we compared the feeding process of the two groups, the study group began oral feeding, complete import feeding, feeding conversion days, and indwelling gastric tube time were lower than the control group, and the data difference was statistically significant (*P* < 0.05). All the data results are shown in Figure 2.

### 3.4. Comparison of Growth and Development

Next, we compared the growth and development of the two groups. The recovery time of birth weight in the study group was lower than that in the control group, the growth of body weight, body length, and head circumference at 14 days in the study group was significantly higher than those in the control group, and the difference was statistically significant (*P* < 0.05). All the data results are shown in Table 2.

### 3.5. Comparison of Feeding Intolerance, Total Enteral Feeding, Jaundice Duration, and Hospitalization Days

Then, we compared the feeding intolerance, the duration of jaundice, and the days of hospitalization between the two groups. The feeding intolerance, the duration of jaundice, and the days of hospitalization in the study group were lower than those in the control group, and the difference was statistically significant (*P* < 0.05). The results of all the data are shown in Table 3.

### 3.6. Comparison of Quality of Life Scores

Finally, we compared the scores of qualities of life between the two groups. Before nursing, there was no significant difference between the two groups (*P* > 0.05). The scores of physiological function, psychological function, and social function in the study group were lower than those in the control group, and the difference was statistically significant (*P* < 0.05). All the data results are shown in Table 4.

The article "Application of Touching Combined with Intelligent Interaction of Voice and Rhythm in Nursing Care of Newborns with Feeding Intolerance and Its Influence on Quality of Life" was retracted in 2023. Reasons: unreliable results or conclusions; concerns about the data; concerns about the peer review; concerns about the citations.

## 4. Discussion

Neonatal feeding intolerance refers to a group of clinical symptoms of abnormal feeding and disorders caused by gastrointestinal dysfunction induced by various disease factors in the neonatal period, which are often characterized by abnormal symptoms of digestive tract, such as vomiting, abdominal distension, and gastric retention [1]. The incidence of neonatal feeding intolerance is high, and the incidence is higher because of lack of gastrointestinal motility. The younger gestational age of the newborn is, the higher the incidence is [10]. Feeding intolerance is defined as (1) vomiting, abdominal distension, or both; (2) an increase in residue, >50% of previous feeding, while the color of gastric residue is also important; and (3) reduction, delay, and interruption of gastrointestinal feeding. Although domestic and foreign scholars have different diagnostic criteria for neonatal feeding intolerance, gastric residual (GRV) is widely used to diagnose neonatal feeding intolerance, but the scope is also different. Furthermore, feeding intolerance is a benign symptom caused by temporary gastrointestinal dysfunction, but some of the symptoms of feeding intolerance have intussusception with the symptoms of other diseases, such as neonatal necrotizing enterocolitis (NEC). Feeding intolerance is the clinical manifestation of NEC as a separate symptom, but it is not clear when feeding intolerance tends to NEC and when it is insufficient [11]. It is necessary for clinicians to judge according to their own clinical experience, and whether it is related to NEC is not very clear. The presence of organic intestinal problems such as left microcolonic syndrome, Hirschsprung's disease, gastric volvulus should be assessed before determining simple feeding intolerance [11, 12].

Touch, also known as massage, is a medical means or adjuvant therapy, which refers to the orderly and rhythmic massage of newborns under the guidance of scientific theory, the method of operation in which comfortable stimuli is transmitted to the central nervous system through the tactile receptors and baroreceptors on the body surface, thus producing positive physiological effects [13]. The concept of touch originated very early and was recorded in ancient times. In 1943, Ribble first used the method of touching to intervene newborns [14]. The results showed that massage could promote the functional development of neonatal respiratory and circulatory system, change neonatal shortness of breath pattern, and maintain effective gas exchange [13]. The study of touching intervention on premature infants was first seen in 1986. Field et al. touched 20 premature infants with an average gestational age of 31 weeks and an average birth weight of 1280 g. It was found that touching was an economical and effective way to promote the growth and development of very low birth weight infants (birth weight < 1500 g) [14]. When preterm infants were placed in the neonatal intensive care unit (NICU) after birth, they often underwent pain stimulation from different sources, which made them in a state of stress for a long time, resulting in a series of physiological and behavioral reactions, such as accelerated heart rate and respiration and decreased oxygen saturation [15]. Touching has a relieving effect on pain, and its mechanism is generally believed that neonatal touching can promote the release of endogenous morphine-like substance *β*-endorphin and play an analgesic role [16]. Meanwhile, touching can increase the concentration of inhibitory neurotransmitter 5-hydroxytryptamine and reduce the tension of vagus nerve, the irritable state of premature infants, enhance their sense of security, sense of satisfaction, and eliminate bad emotions in order to achieve the purpose of relieving pain [16]. By comparing the crying time and quiet sleep time of newborns collecting plantar blood before and after touching intervention, it was found that touching can not only reduce the response to pain stimulation, shorten the crying time, but also prolong the quiet sleep time [17]. Combined with the results of this study, there was no significant difference in feeding performance between the two groups before nursing (*P* > 0.05). After nursing, the feeding rate, milk intake ratio, and proficiency of the two groups increased; and the feeding rate, milk intake ratio, and proficiency of the study group were better than those of the control group. In terms of the feeding process of the two groups, the days of oral feeding, complete import feeding, feeding conversion, and indwelling gastric tube in the study group were lower than those in the control group, and the difference was statistically significant. Touch massages are able to make them feel comfortable, weaken the nervous reaction, stimulate the brain, excite the vagus nerve, promote gastrointestinal peristalsis, accelerate gastric emptying, increase the secretion and activity of gastrointestinal hormones, and facilitate digestion and absorption of nutrients [18, 19].

The article "Application of Touching Combined with Intelligent Interaction of Voice and Rhythm in Nursing Care of Newborns with Feeding Intolerance and Its Influence on Quality of Life" was retracted in 2023. Reasons: unreliable results or conclusions; concerns about the data; concerns about the peer review; concerns about the citations.

Since the 21st century, intelligent voice interaction devices are more and more applied in human daily life. The new generation of products that integrate voice interaction elements into common devices in daily life is also emerging one after another, such as voice input integrated on smart mice and voice input methods on mobile phones. Technology such as sound wave extraction is also a factor that cannot be ignored, which is also part of the reason that hinders the development of the field of voice interaction [20]. If a voice interaction device can communicate like humans, then it must be a device that subverts the field of voice interaction, or a great invention [21]. Although there are no such intelligent interactive devices at present, with the continuous innovation in the era of AI, there will always be real voice interactive devices [22–24].

The application of intelligent interaction technology based on voice rhythm is more convenient than touch screen and keystroke and has the advantage of low threshold, so it does not have to rely on users' digital information foundation and computer professional knowledge [25]. As a result, these voice assistants provide new opportunities for different groups of people, including individuals who are not interested in or unable to use traditional computing devices such as computers and smartphones [26, 27]. Combined with the results of this study, in terms of the growth and development of the two groups, the time for the recovery of birth weight in the study group was lower than that in the control group; and the growth of body weight, body length, and head circumference at 14 days in the study group were higher than those in the control group. The feeding intolerance, the duration of jaundice, and the days of hospitalization in the study group were lower than those in the control group. Moreover, the feeding intolerance, the duration of jaundice, and the days of hospitalization in the study group were lower than those in the control group. Finally, we compared the scores of qualities of life between the two groups. Before nursing, there was no significant difference between the two groups (*P* > 0.05). The physiological function, psychological function, and social function of the study group were lower than those of the control group (*P* > 0.05). The physiological function, psychological function, and social function of the study group were lower than those of the control group. The analysis shows that although developmental nursing strategies have been introduced in pediatrics in the past decade to reduce the stimulation of external stressors to newborns, the impact of sound exposure reduction on newborns has not been paid attention to by medical staff. At present, studies on MSS are mainly related to the effects of MSS on neonatal vital signs, feeding, growth, development, and cognitive behavior, but there is still a lack of unified operating standards. The intelligent interaction technology of phonetic rhythm is used in the nursing of neonatal feeding intolerance. Newborns are stimulated by phonological sounds, including voice, song, and heartbeat. A series of interventions have a positive impact on the physiology, psychology, and behavior of newborns [28, 29]. Neonatal feeding intolerance often requires more care from nurses, and this stage is a key sensitive period for neonatal brain maturity and neural development. Newborns are exposed to a number of stressors, including pain stimuli, bright light, and noise stimuli. In addition, the newborn is also separated from the mother prematurely, and the mother-infant separation delays the establishment of the postpartum mother-child relationship, which hinders the mother's care of the baby and affects the growth of the newborn. Phonetic rhythm and other sensory activities (such as touch, light, and smell) can stimulate the neonatal sensory system and contribute to its growth and development [30, 31]. This study may also have drawbacks such as poor sample representation, erroneous control selection, and recall bias in exposure history. However, in order to obtain reliable results, we did our best to avoid them during the study.

The article "Application of Touching Combined with Intelligent Interaction of Voice and Rhythm in Nursing Care of Newborns with Feeding Intolerance and Its Influence on Quality of Life" was retracted in 2023. Reasons: unreliable results or conclusions; concerns about the data; concerns about the peer review; concerns about the citations.

Conclusively, the application of touch combined with phonetic rhythm intelligent interaction technology in the nursing of neonatal feeding intolerance can promote the faster development and maturity of neonatal gastrointestinal function, facilitate gastrointestinal motility, shorten the time of parenteral nutrition in newborns, faster to achieve total enteral feeding, and promote neonatal growth and development, so as to shorten hospital stay, improve neonatal gastrointestinal feeding tolerance, and improve the quality of life.

## Figures and Tables

**Figure 1:** (a) Comparison of feeding performance between two groups of patients before nursing. (b) Comparison of feeding performance between two groups of patients after.

**Figure 2:** Comparison of feeding process between two groups of patients.

**Table 1:** Comparison of general data of two groups of patients.

Group	Control group (*n* = 70)	Research group (*n* = 70)	*t*/*χ*^2^	*P*
Gestational age (weeks)	34.81 ± 4.12	34.86 ± 4.13	0.071	0.942
Gender (male/female)	43/27	41/29	0.158	0.690
Delivery mode				
Cesarean section	49 (70.00)	47 (67.14)	0.132	0.715
Vaginal delivery	21 (30.00)	23 (32.86)		
Birth weight (g)	1853.75 ± 53.96	1859.74 ± 56.83	0.639	0.523
Head circumference	30.86 ± 1.91	30.63 ± 1.43	0.806	0.421
Body length	48.95 ± 2.44	48.86 ± 2.45	0.217	0.827
Apgar scoring	8.95 ± 0.33	8.99 ± 0.38	0.664	0.507

**Table 2:** Comparison of growth and development between the two groups of patients [±*s*].

Group	Number of cases	Restore birth weight (d)	Body mass increase at 14 days (g)	Body length gain at 14 days (cm)	The head circumference increased at 14 days (cm)
Control group	70	9.58 ± 0.36	24.92 ± 2.65	1.48 ± 0.54	0.72 ± 0.21
Research group	70	8.10 ± 0.54	29.84 ± 2.45	2.59 ± 0.34	1.94 ± 0.21
*t*		19.079	11.405	14.553	34.269
*P*		<0.01	<0.01	<0.01	<0.01

The article "Application of Touching Combined with Intelligent Interaction of Voice and Rhythm in Nursing Care of Newborns with Feeding Intolerance and Its Influence on Quality of Life" was retracted in 2023. Reasons: unreliable results or conclusions; concerns about the data; concerns about the peer review; concerns about the citations.

**Table 3:** Comparison of feeding intolerance, total enteral feeding, jaundice duration, and hospitalization days between the two groups.

Group	Number of cases	Duration of feeding intolerance (d)	Time to reach whole intestinal feeding (d)	Duration of jaundice (d)	Days of hospitalization (d)
Control group	70	8.85 ± 2.05	12.94 ± 2.45	6.56 ± 1.26	17.83 ± 1.45
Research group	70	7.18 ± 1.21	10.85 ± 1.54	4.56 ± 1.45	15.59 ± 1.56
*t*		5.869	6.042	8.710	8.799
*P*		<0.01	<0.01	<0.01	<0.01

**Table 4:** Comparison of quality of life scores between the two groups before treatment.

Group	Number of cases	Physiological function		Psychological function		Social function	
		Before nursing	After nursing	Before nursing	After nursing	Before nursing	After nursing
Control group	70	15.84 ± 4.91	13.86 ± 2.95^a^	16.94 ± 3.91	14.85 ± 4.86^a^	18.82 ± 3.95	16.37 ± 2.81^a^
Research group	70	15.96 ± 4.52	11.84 ± 2.91^b^	16.95 ± 3.86	12.81 ± 1.85^b^	18.84 ± 3.55	12.84 ± 3.81^b^
*t*		0.098	2.670	0.009	2.148	0.020	4.084
*P*		0.921	0.009	0.992	0.035	0.983	<0.01

Note: the control group before and after nursing, ^a^*P* < 0.05; the study group before and after nursing, ^b^*P* < 0.05.

## Data Availability

No data were used to support this study.
